This article has been retracted.

# HDAC4 depletion ameliorates IL‐13‐triggered inflammatory response and mucus production in nasal epithelial cells via activation of SIRT1/NF‐κB signaling

**DOI:** 10.1002/iid3.692

**Published:** 2022-10-11

**Authors:** Hangyu Xu, Lingjun Wang, Huaqun Chen, Hefei Cai

**Affiliations:** ^1^ Department of Otolaryngology, Taizhou Central Hospital Taizhou University Hospital Taizhou Zhejiang China; ^2^ Department of General Practice, Taizhou Central Hospital Taizhou University Hospital Taizhou Zhejiang China; ^3^ Department of Geriatrics, Taizhou Central Hospital Taizhou University Hospital Taizhou Zhejiang China; ^4^ Department of Pediatrics, Taizhou Central Hospital Taizhou University Hospital Taizhou Zhejiang China

**Keywords:** allergic rhinitis, HDAC4, inflammatory response, MUC5AC, SIRT1/NF‐κB signaling

## Abstract

**Introduction:**

Allergic rhinitis (AR) is frequently known as a chronic respiratory disease with a global high prevalence. The pivotal roles of histone deacetylase 4 (HDAC4) in multiple human diseases have been underlined by numerous studies. Nevertheless, whether HDAC4 is implicated in AR remains to be elaborated. The objective of the current study is to clarify the impacts of HDAC4 on AR.

**Methods:**

First, human nasal epithelial cells (hNECs) were pretreated by interleukin‐13 (IL‐13). HDAC4 expression in hNECs with the presence or absence of IL‐13 treatment was tested by quantitative reverse‐transcription polymerase chain reaction (RT‐qPCR) and western blot. Following, after HDAC4 was depleted, levels of histamine, Immunoglobulin E (IgE) and inflammatory factors were analyzed by ELISA assay. Then, Mucin‐5AC (MUC5AC) expression was examined through RT‐qPCR, western blot, and IF assay. Western blot was to analyze the expression of sirtuin 1 (SIRT1)/nuclear factor‐kappaB (NF‐κB) signaling‐related proteins. After IL‐13‐induced hNECs were cotransfected with HDAC4 interference plasmids and SIRT1 inhibitor EX527, the functional experiments above were conducted again.

**Results:**

The experimental data in this study presented that HDAC4 expression was increased in IL‐13‐induced hNECs. Silencing of HDAC4 cut down the levels of histamine, IgE and inflammatory factors and the expression of MUC5AC. Additionally, knockdown of HDAC4 led to the activation of SIRT1/NF‐κB signaling. Further, the downregulated levels of histamine, IgE and inflammatory factors and the expression of MUC5AC imposed by HDAC4 interference were all reversed by EX527.

**Conclusions:**

In short, HDAC4 inhibition activated SIRT1/NF‐κB signaling to mitigate inflammatory response and mucus production in IL‐13‐treated nasal epithelial cells in AR.

## Graphical abstract

Allergic rhinitis (AR) is frequently known as a chronic respiratory disease with global high prevalence. The pivotal roles of histone deacetylase 4 (HDAC4) in multiple human diseases have been underlined by numerous studies. Our paper is the first to explore the role of HDAC4 in AR and the mechanism involved. We concluded that HDAC4 inhibition activated SIRT1/NF‐κB signaling to mitigate inflammatory response and mucus production in interleukin‐13‐treated nasal epithelial cells in AR.

## 1 INTRODUCTION

Allergic rhinitis (AR) is referred to as an upper airway disease, the emergence of which is associated with abnormal immune responses to allergens including dust, pollen, mold, or pet hair in the air.^1^, ^2^ The primary clinical manifestations involving rhinocnesmus, sneezing, rhinobyon, and rhinorrhea may be ascribed to noninfectious inflammation of the nasal mucosa in most cases.^3^, ^4^ As a global public disease, it has been estimated that the incidence rate of self‐reported AR is around 2%–25% in children, and the confirmed rate of AR in adults in Europe varies from 17% to 28.5%.^5^ Meanwhile, morbidity is rising sharply in recent decades as Brozek et al. have suggested.^5^ In addition to its serious impact on life quality, work efficiency, family and socioeconomic burden,^6^ AR is also well documented to be a risk factor for asthma.^7^ To date, therapies based on anti‐inflammatory, antihistamines, antileukotrienes agents remain major options for AR therapy in spite of low therapeutic effects attributed by severe side effects.^8^, ^9^ Considering that it is imperative to develop novel therapeutic targets for AR.

Histone deacetylases (HDACs) are a family of enzymes implicated in the homeostasis of histone acetylation.^10^ A large body of literature has consistently shown that HDACs are promising targets for reversion of abnormal epigenetic changes to halt the course of human diseases, such as cancers, cardiovascular and metabolic diseases and so on.^11^, ^12^, ^13^ HDAC4, a member of the class IIa HDACs, has been proposed to be engaged in a large quantity of cellular and epigenetic processes.^14^ Considerable research efforts have been devoted to the significance of HDAC4 in ischemic stroke,^15^ nasopharyngeal carcinoma,^16^ hepatocellular carcinoma,^17^ and so forth. Notably, The expression levels of HDAC2 and HDAC4 are elevated in chronic sinusitis with nasal polyps.^18^ Nasal polyps are associated with chronic inflammation of nasal sinus mucosa, and antibiotics can inhibit the expression levels of HDAC2 and HDAC4, thus inhibiting chronic inflammation.^19^ There has been increasing awareness that HDAC4 stimulates inflammatory response to aggravate the progression of asthma.^20^, ^21^ Therefore, we speculate whether HDAC4 plays an important role in chronic inflammation and thus regulates the progression of AR disease.

STRING database (https://cn.string-db.org/) predicted that there is a potential interaction between HDAC4 and SIRT1. SIRT1, an NAD(+)‐dependent deacetylase, is a negative regulator of NF‐κB pathway via decreasing the transcriptional activity of NF‐κB.^22^ It is intensively acknowledged that SIRT1/NF‐κB signaling is capable of regulating inflammation and metabolic disorders.^22^ More importantly, Yuan et al. have illuminated that SIRT1 plays a protective role in murine allergic rhinitis through inactivation of HMGB1/TLR4 pathway.^23^ Huang et al have revealed that SIRT1/Nrf2 signaling modulates the inflammation and mucus formation in human nasal epithelial cells following IL‐13 treatment.^24^ However, it has not been reported whether HDAC4 regulates SIRT1 and its downstream pathways in AR.

Therefore, the objective of the current study is to clarify the impacts of HDAC4 on AR and exploring the novel regulatory mechanism of HDAC4/SIRT1/NF‐κB signaling in AR.

## 2 MATERIALS AND METHODS

### 2.1 Cell culture and treatment

hNECs procured from PromoCell GmbH were grown in RPMI‐1640 medium (Haoranbio) accompanied with the addition of 10% FBS (Biologic Industries) and 1% penicillin/streptomycin at 37°C under humidified air with 5% CO_2_. Then, hNECs were administrated by IL‐13 (10 ng/ml; PeproTech, Inc.) for 24 h to mimic an in vitro model of AR,^25^ regarding the non‐IL‐13 hNECs as a negative control group (Control). Additionally, hNECs were pretreated with SITR1 inhibitor EX527 (20 μM; Selleck Chemicals) for 24 h before IL‐13 exposure.^26^

### 2.2 Reverse transcription‐quantitative PCR (RT‐qPCR)

Total RNA was prepared from hNECs by using of TRIzol (Molecular Research Center Inc.) and cDNA conversion was conducted by virtue of Superfast M‐MLV1 reverse transcriptase (Bioswamp). qPCR was performed using SYBR® Green PCR master mix (Bio‐Rad Laboratories, Inc.) in the Agilent MX3000p Real‐Time PCR system (Agilent Technologies, Inc.) as per the manufacturer's protocol under the following conditions: denaturation at 95°C for 5min, followed by 40 cycles of 95°C for 10 s and 60°C for 30 s. The alternations in relative messenger RNA (mRNA) levels were determined using the 2^‐∆∆Cq^ method.^27^ GAPDH was employed to normalize the relative mRNA levels.

### 2.3 Cell transfection

HDAC4 small interfering RNAs (si‐HDAC4#1/2) generated by Takara Biotechnology were to knockdown HDAC4 expression, referring to si‐NC as a small interfering RNA negative control. Lipofectamine™ 3000 (Takara) was adopted in line with the manufacturer's protocol. Cells were collected for follow‐up experiments at 48 h posttransfection.

### 2.4 Enzyme‐Linked immunosorbent assay (ELISA)

With the employment of ELISA kits from Abcam, the levels of histamine (cat. no. ab213975), IgE (cat. no. ab195216), Granulocyte‐macrophage colony‐stimulating factor (GM‐CSF; cat. no. ab174448), eotaxin (cat. no. ab100509), interleukin‐1 beta (IL‐1β; cat. no. ab229384) and interleukin 6 (IL‐6; cat. no. ab178013) were measured in accordance with the standard protocol. A microplate reader (Biotek) was utilized to read the optical density values at 450 nm.

### 2.5 Immunofluorescent staining

After immobilization with 4% paraformaldehyde and permeabilization with 0.5% Triton X‐100, hNECs were cultivated with MUC5AC (cat. no. #61193; 1:400; Cell Signaling Technology) antibody overnight at 4°C. Fluorochrome‐labeled anti‐rabbit secondary antibody (cat. no. ab150077; 1:400; Abcam) was added for 1 h of incubation after washed with phosphate‐buffered saline. Cell nuclei were stained with DAPI (Koritai Biotechnology) and images were captured using a fluorescence microscope (Leica Microsystems, Inc.).

### 2.6 Western blot

With the application of BCA protein assay kit (Pierce Chemical), the prepared protein samples with the aid of Protein extraction kit was quantified. Afterwards, 10% sodium dodecyl sulfate‐polyacrylamide gel electrophoresis was adopted to divide and shift protein samples to polyvinylidene difluoride membranes (Sigma). Incubation in 5% skim milk for half an hour was to impede nonspecific binding. Subsequently, the membranes were probed with primary antibodies including anti‐HDAC4 (cat. no. ab235583; 1:1000; Abcam), anti‐MUC5AC (cat. no. ab198294; 1:20000; Abcam), anti‐SIRT1 (cat. no. ab189494; 1:1000; Abcam), anti‐phosphorylated (p)‐NF‐κB (cat. no. ab247871; 1:1000; Abcam), anti‐NF‐κB (cat. no. ab32360; 1:1000; Abcam), and anti‐GAPDH (cat. no. ab9485; 1:2500; Abcam) at 4°C overnight. The membranes were incubated with horseradish peroxidase (HRP)‐linked anti‐rabbit (cat. no. ab6721; 1:2000; Abcam) secondary antibody on the following day. The ECL detection system (Millipore, WBKLS0100) was utilized to visualize the protein bands and band intensity was determined on Image Lab™ Software (Bio‐Rad, Shanghai, China). GAPDH was used as a loading control.

### 2.7 Statistical analysis

All statistical analyses were executed using GraphPad Prism 8 software (GraphPad Software, Inc.) and continuous variables were displayed as mean ± standard deviation (SD) from three independent experiments. Student's *t*test was used for comparisons between two groups while one‐way analysis of variance followed by Turkey's test was applied for comparisons among multiple groups. A *p* value under .05 was denoted as statistically significant.

## 3 RESULTS

### 3.1 HDAC4 displays elevated expression in IL‐13‐induced hNECs

To identify the role of HDAC4 in AR, HDAC4 expression was tested by RT‐qPCR and western blot in hNECs following treatment with IL‐13. As exhibited in Figure 1, HDAC4 expression was noted to be increased in IL‐13‐treated hNECs relative to the Control group. Briefly, IL‐13 treatment enhanced HDAC4 expression in hNECs.

**Figure 1:** HDAC4 displays elevated expression in IL‐13‐induced hNECs. RT‐qPCR and western blot ascertained HDAC4 expression in hNECs with the presence or absence of IL‐13 treatment. HDAC4, histone deacetylase 4; IL‐13, interleukin‐13; RT‐qPCR, quantitative reverse‐transcription polymerase chain reaction

### 3.2 Silencing of HDAC4 suppresses IL‐13‐evoked inflammation in hNECs

To study the role of HDAC4 in AR, HDAC4 was knocked down by transfection of HDAC4 interference plasmids and the interference efficacy was examined through RT‐qPCR and western blot. Moreover, it was discovered that HDAC4 expression was remarkably cut down in the si‐HDAC4#1/2 group in comparison with the si‐NC group and si‐HDAC4#2 possessed a better interference efficiency (Figure 2A), therefore si‐HDAC4#2 was selected for the subsequent assays. Through ELISA assay, it was observed that IL‐13 prominently increased the contents of histamine and IgE while depletion of HDAC4 reduced the contents of histamine and IgE (Figure 2B). Besides, the results from detection of inflammatory factors including GM‐CSF, eotaxin, IL‐1β, and IL‐6 also implied that HDAC4 downregulation lessened IL‐13‐induced levels of GM‐CSF, eotaxin, IL‐1β and IL‐6 in hNECs (Figure 2C). To sum up, inhibition of HDAC4 alleviated hNECs inflammation following IL‐13 treatment.

**Figure 2:** Silencing of HDAC4 suppresses IL‐13‐evoked inflammation in hNECs. (A) RT‐qPCR and western blot analysis of the interference efficacy of HDAC4‐targeted siRNAs. (B) Levels of histamine and IgE were detected by ELISA assay. (C) ELISA assay examined GM‐CSF, eotaxin, IL‐1β and IL‐6 levels. HDAC4, histone deacetylase 4; IL‐13, interleukin‐13; IgE, Immunoglobulin E; IL‐1β, interleukin‐1 beta; IL‐6, interleukin 6; GM‐CSF, granulocyte‐macrophage colony‐stimulating factor; RT‐qPCR, quantitative reverse‐transcription polymerase chain reaction

### 3.3 HDAC4 deficiency attenuates mucus production in IL‐13‐treated hNECs

To further elaborate the effects of HDAC4 on mucus production in AR, the expression of MUC5AC, a major component of mucus, was determined. RT‐qPCR and western blot analyzed that MUC5AC expression at mRNA level and protein level was increased in IL‐13‐exposed hNECs and was distinctly declined when HDAC4 was downregulated (Figure 3A). As expected, IF assay also uncovered that the upregulated MUC5AC expression due to IL‐13 treatment was lessened by HDAC4 silencing (Figure 3B). Overall, shortage of HDAC4 inhibited IL‐13‐stimulated mucus production in hNECs.

**Figure 3:** HDAC4 deficiency attenuates mucus production in IL‐13‐treated hNECs. (A) RT‐qPCR and western blot analysis of MUC5AC expression. (B) MUC5AC expression was further tested by IF assay. HDAC4, histone deacetylase 4; IL‐13, interleukin‐13; MUC5AC, Mucin‐5AC; RT‐qPCR, quantitative reverse‐transcription polymerase chain reaction

### 3.4 HDAC4 knockdown inactivates the SIRT1/NF‐κB signaling

Interestingly, western blot analyzed that IL‐13 treatment cut down the protein level of SIRT1 and increased the protein level of p‐NF‐κB. After HDAC4 was silenced, SIRT1 protein level was enhanced and p‐NF‐κB protein level was reduced in IL‐13‐induced hNECs (Figure 4). These results above indicated that HDAC4 was a positive regulator of SIRT1/NF‐κB signaling.

**Figure 4:** HDAC4 knockdown inactivates the SIRT1/NF‐κB signaling. Western blot analyzed the protein levels of SIRT1, p‐NF‐κB, and NF‐κB. HDAC4, histone deacetylase 4; IL‐13, interleukin‐13; NF‐κB, nuclear factor‐kappaB; p‐NF‐κB, phosphorylated nuclear factor‐kappaB; SIRT1, sirtuin 1

### 3.5 SIRT1 inhibitor EX527 reverses the impacts of HDAC4 depletion on IL‐13‐primed hNECs

More intriguingly, the upregulated SIRT1 protein level and the downregulated p‐NF‐κB protein level imposed by HDAC4 interference were both restored after the addition of SIRT1 inhibitor EX527 (Figure 5A). At the same time, it turned out that the declined activities of histamine, IgE, GM‐CSF, eotaxin, IL‐1β and IL‐6 in IL‐13‐insulted hNECs on account of HDAC4 deficiency were all enhanced again following treatment with EX527 (Figure 5B,C). In addition, the experimental results from RT‐qPCR, western blot analysis and IF assay revealed that EX527 reversed the diminished MUC5AC expression in IL‐13‐treated hNECs caused by silencing of HDAC4. Taken together, the impacts of HDAC4 knockdown on IL‐13‐exposed hNECs were countervailed by EX527.

**Figure 5:** SIRT1 inhibitor EX527 reverses the impacts of HDAC4 depletion on IL‐13‐primed hNECs. (A) Western blot analyzed the protein levels of SIRT1, p‐NF‐κB, and NF‐κB. (B) Levels of histamine and IgE were detected by ELISA assay. (C) ELISA assay examined GM‐CSF, eotaxin, IL‐1β, and IL‐6 levels. (D) RT‐qPCR and western blot analysis of MUC5AC expression. (E) MUC5AC expression was further tested by IF assay. GM‐CSF, granulocyte‐macrophage colony‐stimulating factor; HDAC4, histone deacetylase 4; IL‐13, interleukin‐13; IgE, Immunoglobulin E; IL‐1β, interleukin‐1 beta; IL‐6, interleukin 6; MUC5AC, Mucin‐5AC; p‐NF‐κB, phosphorylated nuclear factor‐kappaB; NF‐κB, nuclear factor‐kappaB; RT‐qPCR, quantitative reverse‐transcription polymerase chain reaction

## 4 DISCUSSION

AR is a kind of allergic airway disorder primarily manifested by allergen‐driven chronic inflammation and mucus hypersecretion of the nasal mucosal tissues.^28^, ^29^ Previous studies have pointed out that the etiology of allergic diseases is closely associated with the imbalance of T helper (Th)1/Th2 cells.^30^ IL‐13 produced by Th 2 cells has been supposed to be overexpressed in the peripheral blood of AR patients.^31^ Moreover, IL‐13 is deemed as a central mediator in AR through allergic inflammation, the stimulation of mucin synthesis and secretion.^32^, ^33^ Accumulating evidence has hinted that hNECs are prone to bring about a range of biologically crucial cytokines in response to inflammatory induction or anaphylactic reaction.^34^, ^35^ Given the findings mentioned above, the inflammatory response and mucus production in IL‐3‐induced hNECs were investigated to ascertain the severity of AR in vitro.

Existing studies have documented that HDAC4 predominantly participates in neurodegenerative diseases, inflammation disorders, and cardiovascular diseases.^36^ Notably, HDAC4 has been found to be apparently upregulated in chronic rhinosinusitis with nasal polyps.^18^, ^19^ Similarly, the data in our study suggested that HDAC4 expression was increased in IL‐13‐treated hNECs. During the process of AR, histamine is an essential mediator released from mast cells through allergic reactions dependent on IgE, an immunoglobulin.^37^ GM‐CSF can strengthen eosinophil survival to provoke allergic nasal inflammation.^38^ Eotaxins are a family of CC chemokines that recruit eosinophils to inflammatory sites.^39^ MUC5AC is a major component of mucus implicated in a series of malignancies as a potential diagnostic, prognostic and therapeutic target.^40^ IL‐13 has been shown to stimulate the production of mucus and inflammatory‐related cytokines including IgE, GM‐CSF, eotaxin, IL‐1β and IL‐6.^24^ Consistent with these findings, it was also proved that IL‐13 treatment markedly elevated the levels of histamine, IgE, GM‐CSF, eotaxin, IL‐1β, IL‐6 and increased the expression of MUC5AC in hNECs. Moreover, insufficiency of HDAC4 distinctly downregulated the levels of histamine, IgE, GM‐CSF, eotaxin, IL‐1β, IL‐6, and cut down MUC5AC expression in IL‐13‐primed hNECs. All these results implied that silencing of HDAC4 protected against inflammatory response and mucus production in AR. The finding was also supported by Wei et al who have demonstrated that KLF5 deacetylated by HDAC4 potentiates the airway inflammation and remodeling in asthma through enhancing Slug and CXCL12 expression^20^ and Lu et al. who have explicated that HDAC4 targeted by miR‐20a‐5p contributes to allergic inflammation in human mast cells.^21^ As reported, SIRT1 is tightly related to the regulation of multiple cellular events, metabolism and mitochondrial homeostasis.^41^, ^42^, ^43^ Several studies have firmly established that high expression of SIRT1 plays a suppressive role in murine allergic rhinitis.^23^, ^44^ Furthermore, Huang et al. have substantiated that SIRT1 activation mitigates inflammation and mucus formation in IL‐13‐insulted hNECs.^24^ NF‐κB signaling is a core pro‐inflammatory signaling relying on NF‐κB activation.^45^ A great deal of evidence has presented the relationship between SIRT1 and NF‐κB signaling. Specifically, SIRT1 directly inactivates NF‐κB signaling by deacetylating the p65 subunit of NF‐κB complex.^22^, ^46^ Of note, SIRT1 promoter has been revealed to be capable of recruiting HDAC4 and SIRT1 expression can be restored after interference of HDAC4.^47^ In line with these findings, the potential interaction between HDAC4 and SIRT1 was predicted by STRING database (https://cn.string-db.org/). Also, the SIRT1/NF‐κB signaling was suppressed in hNECs following IL‐13 treatment, as evidenced by the downregulated SIRT1 protein level and the upregulated p‐NF‐κB protein level in IL‐13‐treated hNECs. Additionally, HDAC4 depletion stimulated the SIRT1/NF‐κB signaling through elevating the protein level of SIRT1 and lessening the protein level of p‐NF‐κB in IL‐13‐induced hNECs. Furthermore, it turned out that the addition of SIRT1 inhibitor EX527 reversed the decreased p‐NF‐κB protein level, histamine, IgE, GM‐CSF, eotaxin, IL‐1β, IL‐6 levels, MUC5AC expression, and the increased SIRT1 protein level due to HDAC4 knockdown.

Our article has certain limitations. We did not verify the conclusions of this paper in animal experiments, so we decided to verify them in the following experiments. In addition, hNECs were used in our experiment, which should be verified in more cell lines. Our research group will also discuss other cell lines in the future.

To sum up, HDAC4 deficiency eased IL‐13‐evoked inflammatory response and mucus production in hNECs in AR via activating SIRT1/NF‐κB signaling. To the best of our knowledge, this study is the first to definitely clarify the interaction between HDAC4 and SIRT1/NF‐κB signaling in IL‐13‐stimulated hNECs, which may provide compelling evidence demonstrating that HDAC4 may be a novel target for reducing inflammation and preventing the progression of AR. However, the effects of HDAC4 on AR in vivo need to be further explored, which is a major limitation of this study.

## AUTHOR CONTRIBUTIONS

Hangyu Xu and Lingjun Wang conceived and designed the study. Huaqun Chen and Hefei Cai performed the experiments. Hangyu Xu and Lingjun Wang analyzed the experimental data. Huaqun Chen and Hefei Cai wrote and revised the manuscript. All authors have read and approved the final manuscript.

## CONFLICT OF INTEREST

The authors declare no conflict of interest.

## CONSENT FOR PUBLICATION

All the authors agreed to be published.

## Data Availability

The analyzed data sets generated during the present study are available from the corresponding author on reasonable request.
